# Profiling and bioinformatics analyses reveal differential circular RNA expression in NK/T-cell lymphoma-associated hemophagocytic syndrome

**DOI:** 10.1042/BSR20201590

**Published:** 2020-09-16

**Authors:** Changfeng Man, Yu Fan, Guangli Yin, Jiayu Huang, Jujuan Wang, Hongxia Qiu

**Affiliations:** 1 Department of Hematology, The First Affiliated Hospital of Nanjing Medical University, Jiangsu Province Hospital, 300 Guangzhou Road, Nanjing, 210029, Jiangsu Province, China; 2 Department of Cancer Institute, Zhenjiang Clinical Medical College of Nanjing Medical University, The Affiliated People’s Hospital of Jiangsu University, 8 Dianli Road, Zhenjiang 212002, Jiangsu Province, China; 3 Department of Geriatric Hematology, The First Affiliated Hospital of Nanjing Medical University, Jiangsu Province Hospital, 300 Guangzhou Road, Nanjing,210029, Jiangsu Province, China

**Keywords:** Circular RNA, Second-generation sequencing, Bioinformatics analysis, NK/T-LAHS, Biomarker

## Abstract

Circular RNAs (circRNAs) may be potential biomarkers or therapeutic targets of hemophagocytic syndrome (HPS) due to their high stability, covalently closed structure and implicated roles in gene regulation. The aim of the present study was to determine and characterize the circRNAs from natural killer (NK)/T-cell lymphoma-associated hemophagocytic syndrome (NK/T-LAHS). CircRNA in NK/T-LAHS and healthy control patient serum were assessed using next-generation sequencing (NGS). One hundred and forty-three differentially expressed circRNAs of which 114 were up-regulated and 29 were down-regulated in NK/T-LAHS patients were identified. Next, Gene Ontology (GO) function and Kyoto Encyclopedia of Genes and Genomes (KEGG) pathway analyses to explore the roles of these circRNAs were utilized, and a microRNA (miRNA) target gene prediction software to predict the interaction of circRNAs and miRNAs was used. Moreover, five circRNAs were then selected as NK/T-LAHS candidate circRNAs which were related to tumors and contained NK/T-LAHS-related miRNA-binding sites. Using real-time PCR, the significant up-regulation of these five circRNAs in NK/T-LAHS patient serum were verified. Together these results show that circRNAs may serve as valuable diagnostic biomarkers of early NK/T-LAHS, with potential therapeutic targets in disease progression.

## Introduction

Hemophagocytic lymphohistiocytosis (HLH), also called hemophagocytic syndrome (HPS), is a potentially life-threatening disease characterized by impaired natural killer (NK) and cytotoxic T-cell function, cytokine storm and overwhelming inflammation [1,2]. Recent studies have demonstrated that hyperbilirubinemia, viral infection, NK/T lymphoma, ferritin, serum β2-microglobulin, and serum fibrinogen predict the survival outcomes of secondary HLH (sHLH) patients [3–6]. However, the prognostic accuracy of these clinical parameters has not been fully verified in patients with sHLH. Novel prognostic biomarkers mirroring different pathophysiological mechanisms need to be identified for individualized risk assessment.

Circular RNA (circRNA) is a novel molecule that is formed by a covalently closed loop with different sizes and sources and represents a class of abundant, stable and widely existing RNA molecules in animals [7,8]. It plays an important role in biological processes (BPs). For example, circRNAs act as microRNA (miRNA) sponges [9], RNA-binding proteins and mRNA ‘magnets’ to guide protein translation [10]. CircRNA interacts with disease-related miRNA through a competitive endogenous RNA (ceRNA) mechanism, and plays an important regulatory role in disease[11,12]. However, the role of circRNA in NK/T-cell lymphoma-related hemophagocytic syndrome has not been determined.

With the continuous development of sequencing technology, RNA-Seq (RNA sequencing) based on a high-throughput platform has become an effective tool for mining and identifying new transcripts. Due to the application of high-throughput RNA sequencing and bioinformatics methods, a large amount of circRNA has been found in human cells. Emerging research evidence shows that many circRNAs are specifically expressed in different cells and are related to the normal physiological development of cells and various diseases [13]. CircRNA is widely expressed in human cells and has high abundance. Most of them are structurally stable and have the characteristics of tissue-specific expression and time-specific expression. Previous studies have reported that circRNA is involved in the regulation of the pathogenesis of many diseases, such as cancer, cardiovascular diseases and autoimmune diseases [14–17]. CircRNA is mainly located in the cytoplasm and has microRNA (miRNA) response elements, which can bind to miRNA to prevent it from binding to mRNA targets, inhibit miRNA function, or participate in the regulation of miRNA reduction activity, thereby playing an important role in diseases [18]. At present, a variety of circRNA is differentially expressed between cancer and normal tissues, indicating that circRNA may be a potential tumor biomarker with potential functions and clinical significance [19–21]. However, there are few studies on the expression profile and function of circRNA in NK/T-LAHS.

In the study, we identified a group of circRNAs with differential expression using next-generation sequencing (NGS) technology and explored the roles of these circRNAs by an miRNA target gene prediction software. With real-time PCR, five selected NK/T-LAHS candidate circRNAs were verified for the significant up-regulation.

## Materials and methods

### Study subjects

From 2018 to 2019, in the Department of Geriatric Hematology, the First Affiliated Hospital of Nanjing Medical University, Jiangsu Province, the serum of 4 NK/T-LAHS patients who did not receive cancer treatment and 4 healthy control serums were collected, each with 200μl. The diagnosis of HLH is established according to the 2004 HLH diagnostic criteria [22]. The diagnosis of NK/T-cell lymphoma met pathological criteria through biopsy samples according to the 2016 revision of the World Health Organization classification of lymphoid neoplasms [23]. The sera from the eight blood samples were separated immediately and stored at −80°C until RNA extraction. Second-generation sequencing technology and real-time PCR were then used for circRNA screening and identification. In this study, all participants informed consent, and were approved by the Ethics Committee of the First Affiliated Hospital of Nanjing Medical University (Reference Number: 2019-SR-446).

### RNA isolation, RNA-sequencing library preparation, and sequencing

Total RNA was extracted from the eight serum samples with TRIzol (Life Technologies, Carlsbad, CA, U.S.A.). The NanoDrop ND-1000 instrument (Thermo Fisher Scientific, Waltham, MA, U.S.A.) was used to evaluate the concentration of each RNA sample. All RNA samples involved in this study met the qualification ratio (1.8-2.1) of OD 260 to OD 280, and met the quality control standards. RNA integrity and gDNA contamination were measured by modified agarose gel electrophoresis. Agilent 2100 Bioanalyzer was used to determine the quality of the test library.

RNA high-throughput sequencing was performed by Cloud-Seq Biotech (Shanghai, China). Briefly, total RNA was used to remove the rRNAs with the NEBNext, rRNA Depletion Kit (New England Biolabs, Inc., Massachusetts, U.S.A.) following the manufacturer’s instructions. RNA libraries were constructed by using the NEBNext® Ultra™ II Directional RNA Library Prep Kit (New England Biolabs, Inc., Massachusetts, U.S.A.) according to the manufacturer’s instructions. Libraries were quality controlled and quantified using the BioAnalyzer 2100 system (Agilent Technologies, Inc., U.S.A.). Library sequencing was performed on an Illumina HiSeq instrument with 150-bp paired end reads. The 10 pM library was transformed into single-stranded DNA molecules, which was captured on an Illumina Flowcell (Illumina, U.S.A.), amplified into clusters *in situ*, and sequenced in 150 cycles with PE mode on an Illumina HiSeq (Illumina HiSeq 4000, U.S.A.) sequencer.

### CircRNA profiling analysis

Paired-end reads were obtained from the Illumina HiSeq 4000 sequencer data and were quality controlled by Q30. Then, 3′ adaptor trimming and removal of low-quality reads were performed by cutadapt software (v1.9.3) [24]. The high-quality trimmed reads were used to analyze circRNAs. The high-quality reads were aligned to the reference genome/transcriptome with STAR software (v2.5.1b) [25], circRNAs were detected and identified with DCC software (v0.4.4) [26], and the identified circRNA were annotated with the circBase database and Circ2Traits [27,28]. EdgeR software (v3.16.5) was used to normalize the data and perform differentially expressed circRNA analysis [29]. The circRNAs that had a fold change value ≥ 2.0 and *P*-values ≤0.05 were designated as being significantly differentially expressed. Gene Ontology (GO) and Kyoto Encyclopedia of Genes and Genomes (KEGG) analyses were performed for the differentially expressed circRNA-associated genes. The interaction network between circRNAs and their downstream miRNAs was constructed by Cytoscape software (v2.8.0) based on data of circRNAs with specific miRNA binding sites and their predicted miRNA partners.

### Quantitative real-time polymerase chain reaction analysis

The qPCR verification of specific circRNA was performed to confirm that the data generated by the sequencing work is reliable. Total RNA obtained from serum with TRIzol (Invitrogen, Carlsbad, CA USA) was used for synthesizing cDNA with the ReverTraAc real-time qPCR kit (Toyobo, Osaka, Japan). First-strand cDNA was used for PCR, which was performed in triplicate with SYBR Green Super Mix (Bio-Rad, Hercules, CA, USA). The specific primers sequences for the 5 upregulated circRNAs used for RT-qPCR are summarized in Table 1.

**Table 1:** The five up-regulated circRNA-specific primer sequences for RT-qPCR

CircRNA ID	Sequence (5′–3′)
chr5:112090570-112137080+	F: AGCGGCAGAATGAAGGTCAA
	R: GCCATCCTTGGCTACCCTTG
chr1:77620134-77635080−	F: GGAAGTGTACGGAAAGTGGA
	R: GGCCATATCATCTGCAAGCATT
chr12:62715245-62749256+	F: GCCTCTGTGGCCTAAGTAAC
	R: CTGGTCTCCTTTTCATCTGGA
chr20:34304662-34320057−	F: GTAAGGAACGGAAGCGAAGT
	R: TCGCCTCTCTTTGCTTCTACT
chr6:56989532-57025950+	F: ACATGGGTGCCAAAAATACTTC
	R: GACGAGCCAGAGTTAAAGCAAC
GAPDH	F: GGCCTCCAAGGAGTAAGACC
	R: AGGGGAGATTCAGTGTGGTG

Abbreviations: F, forward; R, reverse.

All reactions were conducted according to the following procedures, 40 PCR cycles (95°C, 10 s; 60°C, 60 s (measure fluorescence)). The fusion curve of PCR products was established as follows: 95°C, 10 s; 60°C, 60 s; and 95°C, 15 s after the amplification reaction, followed by slowly heating from 60 to 99°C (the ramp up rate of the instrument was 0.05°C/s). Each sample was assayed three times.

### Bioinformatics analysis and target prediction

The interaction between circRNA and miRNAs was analyzed and predicted using TargetScan and miRanda database, where they might act as sponges. Based on its related mRNA, Gene Ontology (http://www.geneongolo-ty.org/) and KOBAS (KEGG Orthology Based Annotation System) are used to assess the function of genes associated with detected differentially expressed circRNAs. Genes associated with differentially expressed circRNA detected. The first 300 circRNA-miRNA interaction networks were drawn using Cytoscape software in order to understand the interactions between circRNAs and miRNAs. Based on the two databases previously described, miRNA response element (MRE) is predicted and explained [30–32].

### Statistical analysis

Statistical analysis was performed using SPSS 19.0 (SPSS Corporation, USA) statistical software package. Student's *t* test was used to compare the two variables of next-generation high-throughput sequencing data for statistical analysis. The differences of FC≥2 or≤0.5 and *P*<0.05 were considered to be statistically significant. Calculate the false discovery rate (FDR) to correct the P value of high-throughput sequencing analysis. In qRT-PCR analysis, the 2(-ΔΔCt) method is used to express the level of each circRNA as a fold change.

## Results

### Profiling of circRNAs in NK/T-LAHS patient sera

We utilized Illumina HiSeq instrument to profile circRNA expression in four NK/T-LAHS serum samples and four healthy control serum samples (Table 2). In the four NK/T-LAHS samples, the total reads were 85833954, 88495030, 79053298 and 86398392, yielding mapped read counts of 61953110, 65427958, 58369924 and 63262850, respectively. For the healthy controls, the read counts were 83389774, 83205550, 86771462 and 82877972, yielding mapped read counts of 47656180, 44744062, 50073200 and 46639532, the total reads respectively **(here to remove)**.

**Table 2:** Summary of reads statistics of NK/T-LAHS and normal control

Sample name	Raw reads	Q30	Clean reads	Clean ratio	Mapped reads	CircRNA number
NK/T-LAHS 1	85833954	90.79%	85454974	99.56%	61953110	1362
NK/T-LAHS 2	88495030	91.36%	88239244	99.71%	65427958	1828
NK/T-LAHS 3	79053298	90.85%	78702788	99.56%	58369924	3301
NK/T-LAHS 4	86398392	90.63%	86143752	99.71%	63262850	818
NC-1	83389774	90.20%	82762386	99.25%	47656180	1187
NC-2	83205550	89.99%	82129898	98.71%	44744062	1542
NC-3	86771462	90.12%	86368674	99.54%	50073200	1390
NC-4	82877972	90.56%	82220232	99.21%	46639532	1646

Abbreviation: NC, normal control.

In total, we were able to identify 11481 different putative circRNAs in these serum samples, of which 2698 were consistent with circRNAs in circBase (http://www.circbase.org) and 42 were documented in the literature. The remaining 8741 are novel circRNAs first identified in this document (Figure 1A). Using the RefSeq database, we annotated the identified circRNAs and found that 2990 contained protein-coding exons, while 4288, 2110, 1126, and 967 circRNAs aligned with introns, antisense, intergenic, and sense overlapping regions of known transcripts, respectively (Figure 1B). The length of the majority of identified exonic circRNAs (2990 total) was under 1500 nucleotides (nt), with the majority being 200–1000 nt (Figure 1C). The chromosome distributions of circRNAs are shown in Figure 1D, with the majority being concentrated on chromosomes 1 and 2.

**Figure 1:** The overall circRNA sequencing (**A**) The source of circRNAs in NK/T-LAHS, 11481 different putative circRNAs in these serum samples were identified, of which 2698 were consistent with circRNAs in circBase, 42 were documented in the literature, and 8741 were novel circRNAs first identified. (**B**) The catalog of circRNAs in NK/T-LAHS, using the RefSeq database, 2990 contained protein-coding exons, while 4288, 2110, 1126, and 967 circRNAs aligned with introns, antisense, intergenic, and sense overlapping regions of known transcripts, respectively. (**C**) The length range of circRNA in NK/T-LAHS, the length of the majority of identified exonic circRNAs (2990 total) was under 1500 nt, with the majority being 200–1000 nt. (**D**) The chromosome distribution of circRNA in NK/T-LAHS, The chromosome distributions of circRNAs with the majority being concentrated on chromosomes 1 and 2.

### Differentially expressed circRNAs in NK/T-LAHS serum

The differential circRNAs between the NK/T-LAHS and normal control groups were determined through fold change and *P*-values (fold change ≥ 2.0; *P*-values ≤0.05) statistical criteria. Finally, of the identified circRNAs, 143 were specifically and significantly differentially expressed in NK/T-LAHS samples. In contrast with those in the normal control group, a total of 114 circRNAs were markedly up-regulated and 29 were significantly down-regulated in the NK/T-LAHS group, as shown by a cluster heatmap (Figure 2A). The most significantly up-regulated and down-regulated circRNAs were chr22:20981567–20981750+ (fold change 219.967531 up; *P*-values <0.05) and hsa_circ_0123217 (fold change 369.5452384 down; *P*-values <0.05), respectively.

**Figure 2:** Differentially expressed circRNAs in NK/T-LAHS (**A**) Cluster heatmap of intersection expressed circRNAs in NK/T-LAHS patients compared with normal controls (NC). In the clustered heatmap identified by NGS, each column represents serum from a patient or a healthy volunteer, each line represents a circRNA. The red lines are up-regulated circRNAs, and the green ones are down-regulated circRNAs. Five up-regulated circRNAs which were verified by real-time qPCR were marked. (**B**) Scatter plot of intersection expressed circRNAs in NK/T-LAHS patients compared with NC. Vertical green lines indicate two-fold (log_2_ scaled) up- or down-regulation, and the horizontal green line indicates a *P*-value of 0.05 (−log_10_ scaled). Red squares represent circRNAs with statistically significant differences in expression. (**C**) Volcano plot of intersection expressed circRNAs in NK/T-LAHS patients compared with NC, differentially expressed circRNAs between NK/T-LAHS and NC are displayed by volcano plots. Vertical green lines indicate two-fold (log_2_ scaled) up or down changes, and the horizontal green line indicates a *P*-value of 0.05 (−log_10_ scaled). Red squares represent circRNAs with statistically significant differences in expression.

Differentially expressed circRNAs between the NK/T-LAHS group and normal controls are displayed by scatter plots (Figure 2B) and volcano plots (Figure 2C). Vertical green lines indicate two-fold (log_2_ scaled) up- or down-regulation, and the horizontal green line indicates *P*-values of 0.05 (−log_10_ scaled). Red squares represent circRNAs with statistically significant differences in expression.

### Functional analysis of target genes

The ‘Gene Ontology’ (http://www.geneontology.org) project provides a controlled vocabulary for describing the attributes of genes and gene products in any organism. The ontology covers three domains: BP, cellular component (CC), and molecular function (MF). The top ten GO terms were identified. ‘Positive regulation of pseudopodium assembly,’ ‘regulation of pseudopodium assembly,’ and ‘pseudopodium assembly’ were the top three BPs (Figure 3A); ‘β-catenin destruction complex,’ ‘complex of collagen trimers,’ and ‘clathrin coat of trans-Golgi network vesicle’ were the top three CCs (Figure 3B); and ‘receptor antagonist activity,’ ‘GTP-Rho binding,’ and ‘hydrolase activity, acting on ether bonds’ were the top three MFs (Figure 3C).

**Figure 3:** GO annotations of expressed circRNAs in NK/T-LAHS (**A**) BPs. (**B**) CCs. (**C**) MFs. GO enrichment analysis was made up of (A) BPs, (B) CCs, and (C) MFs. The top ten predicted functions of the source gene regulated by 114 up-regulated circRNAs in serum from patients with NK/T-LAHS were explored by GO analysis. Fold enrichment indicated the regulated extent of the predicted functions by up-regulated circRNAs in NK/T-LAHS patients compared with normal controls (NC).

When we performed a KEGG pathway analysis, a total of 21 pathways were enriched in these circRNAs. The top ten pathways were identified (Figure 4A). Insulin signaling pathways up-regulated by circRNA in NK/T-LAHS (Figure 4(b)), endometrial cancer (Figure 4(c)), and hippopotamus signaling (Figure 4(d)) are the three most important signal transduction pathways. These three most important signaling pathways are related to the expression of GSK-3β, which plays a crucial role in the pathogenesis of NK/T-LAHS. These pathway analyses indicated that up-regulated circRNAs in the serum of NK/T-LAHS patients may have substantial implications for this disease.

**Figure 4:** KEGG pathway annotations of expressed circRNAs in NK/T-LAHS (**A**) The top ten KEGG pathway analysis enriched in circRNAs. (**B**) Insulin signaling pathway. (**C**) Endometrial cancer. (**D**) Hippo signaling pathway, insulin signaling pathway, endometrial cancer. Hippo signaling pathways regulated by the up-regulated circRNAs in NK/T-LAHS. The KEGG analysis revealed 21 signaling pathways related to the 114 up-regulated circRNAs in patients with NK/T-LAHS. (B) Insulin signaling pathway, (C) endometrial cancer pathway, and (D) Hippo signaling pathways were connected with expression of GSK-3β, which played a crucial role in pathogenesis of NK/T-LAHS.

### circRNA-targeted miRNA–gene network generation

Among the 143 differentially expressed circRNAs, we selected 5 circRNAs for further study. They were chr5:112090570-112137080+ (hsa_circ_0073586), chr1:77620134-77635080− (hsa_circ_0114150), chr12:62715245-62749256+ (hsa_circ_0027353), chr20:34304662-34320057− (hsa_circ_0115056), chr6:56989532-57025950+ (hsa_circ_0131996). These five circRNAs had increased differential expression in NK/T-LAHS compared with normal samples. In addition, these 5 circRNAs all contain miRNA targets related to NK/T-LAHS.Therefore, we conclude that these 5 circRNAs may be closely related to NK/T-LAHS. Since circRNA can have many miRNA targets, we summarize the top 5 sites of each circRNA in (Table 3). The figure shows that circRNA interacts with miRNA in many ways. (Figure 5).

**Figure 5:** The interaction network between differentially expressed circRNAs and miRNAs in NK/T-LAHS Five up-regulated circRNAs were selected for validation (yellow), and are displayed in a network diagram. The graph shows that circRNAs interacted with miRNAs in numerous ways. The top five miRNAs regulated by each circRNA are shown (green). Circles indicate circRNAs and arrows represent miRNAs.

**Table 3:** Predicted miRNAs for the five selected differentially expressed circRNAs linked to NK/T-LAHS

CircRNA ID	miRNA	miRNA	miRNA	miRNA	miRNA
chr5:112090570-112137080+	hsa-miR-6821-3p	hsa-miR-6728-3p	hsa-miR-6800-3p	hsa-miR-337-5p	hsa-miR-7-5p
chr1:77620134-77635080−	hsa-miR-215-3p	hsa-miR-485-3p	hsa-miR-5089-5p	hsa-miR-1302	hsa-miR-593-3p
chr12:62715245-62749256+	hsa-miR-29b-1-5p	hsa-miR-6843-3p	hsa-miR-7-5p	hsa-miR-1299	hsa-miR-6876-3p
chr20:34304662-34320057−	hsa-miR-138-1-3p	hsa-miR-425-3p	hsa-miR-183-5p	hsa-miR-6841-3p	hsa-miR-5009-5p
chr6:56989532-57025950+	hsa-miR-4268	hsa-miR-6514-3p	hsa-miR-146a-3p	hsa-miR-6741-5p	hsa-miR-1273d

### Verification of selected circRNAs

This study first evaluated circRNA in the serum of NK/T-LAHS and healthy control patients through next-generation high-throughput sequencing. Then qRT-PCR was used to detect the circRNA expression levels of the serum samples of ten NK/T-LAHS patients and ten healthy volunteers to verify the accuracy of the sequencing data.In addition, GO, Pathway analysis and circRNA-miRNA network analysis were also carried out to preliminarily explore the biological functions of these circRNAs in the occurrence and development of HPS. We selected five circRNAs as NK/T-LAHS candidate circRNAs associated with tumors and containing NK/T-LAHS-related miRNA binding sites to verify NGS data. They were found to be consistent between RNA-seq and qRT-PCR, and circRNA in the serum of NK/T-LAHS patients was up-regulated, suggesting its potentially important clinical significance (Figure 6).

**Figure 6:** Five up-regulated circRNAs in patients with NK/T-LAHS compared with normal controls The serum from ten NK/T-LAHS patients and ten healthy volunteers were used for verification by real-time qPCR on the basis of circRNAs sequencing. The relative expression of the five up-regulated circRNAs in serum from NK/T-LAHS compared with NC were verified by real-time qPCR. hsa_circ_0073586 (*P*=0.001), hsa_circ_0114150 (*P*=0.000), hsa_circ_0027353 (*P*=0.003), hsa_circ_0115056 (*P*=0.000) and hsa_circ_0131996 (*P*=0.036) exhibited the same growing trend toward the sequencing results. *P<0.05, ** *P*<0.01, and *** *P*<0.001.

## Discussion

Hematological malignancies are the most common risk factors for HLH. Most of them have a poor prognosis, and LAHS patients have the worst prognosis. Early diagnosis of the underlying conditions, especially NK/T-LAHS, may lead to better outcomes [33,34]. At present, there are no biomarkers of NK/T-LAHS sensitive enough for diagnostic purposes. Therefore, it is necessary to identify new biomarkers and explore their functions. In this study, when looking for biomarkers related to disease progression, a new useful marker for early diagnosis of LAHS was identified. This marker can sensitively and effectively diagnose early NK / T-LAHS, which will be confirmed in further studies.

Recent studies have revealed that circRNAs are involved in gene regulation during the transcriptional and posttranscriptional stages [35]. CircRNA can regulate the expression of targeted genes by interacting with RNA binding proteins [9]. These circRNAs can perform unique functions. Because they can be detected at higher levels in exosomes. Therefore, they can be good biomarkers for cancer diagnosis [36].

Many studies have proved that circRNAs are involved in the pathogenesis of various diseases and are potential biomarkers [14,37–39]. Some research results have shown that circRNAs are moderately effective assistant diagnostic biomarkers for lymphoma. However, to date, few studies have assessed these molecules as biomarkers for NK/T-LAHS. Mei M et al. found that circCDYL is highly expressed in the plasma of MCL (mantle cell lymphoma) patients, and inhibiting circCDYL can inhibit the proliferation of MCL cells, suggesting that circCDYL may be a potential diagnostic biomarker [40]. Hu Y et al. studied the expression of circRNA in diffuse large B-cell lymphoma (DLBCL) and found that circ-APC was down-regulated in DLBCL tissues, cells and plasma. This indicates that circ-APC is a new type of proliferation inhibitor. Restoring Circ-APC expression may be a promising treatment for patients with DLBCL [41]. Deng et al. showed that circ-LAMP1 was overexpressed in T-cell lymphoblastic lymphoma (T-LBL) tissues and cell lines and modulated cell growth and apoptosis by regulating the miR-615-5p/DDR2 pathway in T-LBL. These findings demonstrated that circ-LAMP1 might be an oncogene in T-LBL, which might be useful in developing promising therapies for T-LBL [42]. Dahl M et al. discovered a new gold standard for circRNA quantification, that is, an enzyme-free digital counting method to summarize the expression of circRNA in B-cell malignancies [43]. However, the functional mechanism of circRNAs in NK/T-LAHS is poorly understood.

Therefore, it is significant to profile the circRNA expression and find new biomarkers, which may help to provide new directions and strategies for the diagnosis and treatment of diseases, and is reasonable to hypothesize that there might be certain circRNAs’ expression styles which were characteristic of NK/T-LAHS. In this study, we compared circRNA expression patterns between NK/T-LAHS and healthy control serum samples using second-generation circRNA sequencing.Through our sequencing work, we were able to identify a large number of specific circRNAs, including many that are not yet available in the circRNA databasess. In addition, in order to explore the full content of circRNA, we described the length and chromosome distribution model of circRNAs in serum of NK/T-LAHS patients.

Progressively, we identified circRNA expression in 143 NK/T-LAHS and control serum samples, most of which were up-regulated in NK/T-LAHS patients, indicating that they may be related to the occurrence and development of NK/T-LAHS. Others have similar views to us. For example, Huang et al. detected bladder urothelial carcinoma and renal clear cell carcinoma and found that circRNA was significantly upregulated [44] and Wang et al. detected the expression of circRNA in the serum of patients with ovarian cancer and found 178 differentially expressed circRNAs, of which 175 were up-regulated and only 3 were down-regulated [15]. However, there are also opposite results. For example, Zheng et al. found significant down-regulation of circRNA in colorectal cancer and gastric cancer [45]. However, there are also different conclusions. For example, Zheng et al. generated RNA sequencing data of ribosome consumption and found that significant circRNA down-regulation was detected in cancer tissues [45]. So far, the functions of most circRNAs have not been well understood, and their expression changes are very common in diseases. The specific role of circRNA in NK/T-LAHS is still uncertain. We use Gene Ontology to analyze the correlation between the expression of circRNA and its linear counterpart [46]. The ontology covers three domains: BP, CC, and MF **(here to remove)**. GO function analysis of the host genes of differentially expressed circRNAs was performed to annotate and predict the function of these circRNAs. KEGG pathway analysis is the process of mapping molecular datasets in genomics, transcriptomics, proteomics, and metabolomics to KEGG pathway maps to explain the biological functions of these molecules. By analyzing the pathways of differentially expressed genes derived from circRNAs, we can infer the pathways in which they participate and their biological functions **(here to remove)**. Through KEGG pathway analysis, we determined that these circRNAs were enriched in pathways including insulin signaling, endometrial cancer, Hippo signaling, basal cell carcinoma, colorectal cancer, PI3K-Akt signaling, prolactin signaling, focal adhesion, ECM–receptor interaction, and regulation of actin cytoskeleton. These pathway analysis methods together emphasize the broad regulatory role that circRNAs can play in the context of some diseases, and circRNAs may affect a variety of cellular functions by changing their regulation. Most Akt substrates are involved in the regulation of cell survival and cell cycle progression. This is the core role of the PI3K/AKT pathway in promoting the progression of human malignant tumors. There have been some reports on the influence of AKT signaling in tumorigenesis and cancer progression [47,48].The relationship between PI3K activity disorder and abnormal proliferation has been fully demonstrated. PI3K activity is related to a series of human tumors, such as breast cancer, lung cancer, melanoma and leukemia. In addition, there is evidence that AKT is a downstream enzyme of PI3K and is also involved in malignant transformation [49]. However, there is no study on PI3K/AKT signaling pathway in NK/T-LAHS. Our study shows that up-regulated circRNA participates in this important signaling pathway, and we still need to further explore how the signaling pathway works and whether it can become a new therapeutic target.

In addition, substantial evidence has suggested that circRNAs can play many significant roles, such as acting as competitive endogenous RNAs to sponge miRNAs efficiently, attenuating or compromising the inhibitory effect of miRNAs on target genes, and modulating protein synthesis accordingly [9,35,50]. CircRNAs can decrease or eliminate the inhibition of miRNAs on target genes and regulate protein synthesis correspondingly [51]. There has been little research on how circRNAs and miRNAs interact in the context of NK/T-LAHS, so we constructed a circRNA-miRNA network for NK/T-LAHS using our sequencing results. Based on miRNA binding site predictions, we selected five significantly up-regulated circRNAs (chr5:112090570-112137080+ (hsa_circ_0073586), chr1:77620134-77635080− (hsa_circ_0114150), chr12:62715245-62749256+ (hsa_circ_0027353), chr20:34304662-34320057− (hsa_circ_0115056) and chr6:56989532-57025950+ (hsa_circ_0131996)) that may be closely related to NK/T-LAHS. We further confirmed that these circRNAs are up-regulated in the serum of NK/T-LAHS patients by qPCR, indicating that these five circRNAs may be potential biomarkers for NK/T-LAHS. All these circRNAs have multiple binding sites for NK/T-LAHS-related miRNAs. For example, hsa-circ_0131996 has an miR-4268 binding site, miR-6514-3p binding site, miR-146a-3p binding site, miR-6741-5p binding site and miR-1273d binding site. Previous studies have reported that miR-142-3p, miR-451, miR-144, miR-143-3p, miR-106b, and miR-101 are up-regulated in HLH and may be associated with the immune/inflammatory response in patients with HLH [52]. Li Wei et al. found that the average level of miR-133 in LAHS was significantly higher than that of HLH related to benign diseases [53]. Bay et al. evaluated the plasma miRNA expression levels in secondary HLH and showed that miR-205-5p and miR-194-5p were up-regulated and miR-30c-5p was down-regulated in HLH, which could be useful plasma biomarkers for HLH [54]. According to reports, circular RNA can act as a microRNA sponge. Recently, circular RNAs have been proposed to accommodate microRNAs and found to be rich in functional miRNA binding sites. Therefore, we predict that hsa_circ_0131996 is a miRNA sponge. We further explored the potential value of these complex circRNA-miRNA networks to explore the causes of disease progression. Our results found a serious dysregulation of circRNA in NK/T-LAHS. In the serum of these patients, most of the detectable circRNA are significantly overexpressed. These new disease-related circular RNAs can be used as new biomarkers for the diagnosis of NK/T-LAHS patients and can provide new insights for various diseases.

The present study had several limitations. The human NK/T-LAHS samples of the present study were only from four patients, and the sample size was too small. Furthermore, identification of differentially expressed circRNAs in subjects with NK/T-LAHS based on RNA-sequencing (RNA-seq) and verification of the circRNA profile by qPCR needs to be conducted in another independent large-size sample cohort. Additionally, because functional validation assays were not included in the present study, the specific mechanisms by which circRNAs may be involved in NK/T-LAHS development were not speculated on. Finally, the role of circRNA in the pathogenesis of the disease has not been explored in this experiment. In the future, we will collect patients' peripheral blood mononuclear cells to detect the expression of circRNA in the cells. The target gene of circRNA is predicted by bioinformatics technology, and the signal pathway of the predicted target gene is verified by dual luciferase report.

In summary, we identified 11481 cirRNAs in human NK/T-LAHS samples. Based on comparisons with current databases, 76% of circRNAs were identified as novel. Further analysis showed that 114 up- and 29 down-regulated circRNAs were distinctly associated with NK/T-LAHS disease. The results suggested that the 143 identified circRNAs might serve as valuable diagnostic biomarkers of early NK/T-LAHS.

## Abbreviations

BP: biological process
CC: cellular component
circCYDL: circular RNA CYDL
circRNA: circular RNA
DDR2: discoidin domain receptor 2
DLBCL: diffuse large B-cell lymphoma
ECM: extracellular matrix
gDNA: genomic DNA
GO: Gene Ontology
GSK-3β: glycogen synthase kinase-3β
HLH: hemophagocytic lymphohistiocytosis
HPS: hemophagocytic syndrome
IL-2R: interleukin-2 receptor
KEGG: Kyoto Encyclopedia of Genes and Genomes
LAHS: lymphoma-associated hemophagocytic syndrome
MCL: mantle cell lymphoma
MF: molecular function
miRNA: microRNA
NGS: next-generation sequencing
NK: natural killer
NK/T-LAHS: NK/T-cell lymphoma-associated hemophagocytic syndrome
OD: optical density
qPCR: quantitative polymerase chain reaction
RT-qPCR: reverse transcription-quantitative polymerase chain reaction
sHLH: secondary HLH
T-LBL: T-cell lymphoblastic lymphoma
